# Triage Nurse-Activated Emergency Evaluation Reduced Door-to-Needle Time in Acute Ischemic Stroke Patients Treated with Intravenous Thrombolysis

**DOI:** 10.1155/2022/9199856

**Published:** 2022-03-03

**Authors:** Xiao Liang, Wenhui Gao, Jiali Xu, Sara Saymuah, Xiaojie Wang, Jing Wang, Wenbo Zhao, Xiurong Xing, Changyuan Wang, Fangyan Liu, Lei Feng, Sijie Li

**Affiliations:** ^1^Department of Emergency, Xuanwu Hospital Capital Medical University, Beijing, China; ^2^Department of Neurology, Xuanwu Hospital Capital Medical University, Beijing, China; ^3^Wayne State University School of Medicine, Detroit, USA; ^4^Department of Neurology, Shenzhen Qianhai Shekou Free Trade Zone Hospital, Shenzhen, China; ^5^Beijing Institute of Brain Disorders, Capital Medical University, Beijing, China; ^6^Beijing Key Laboratory of Hypoxic Conditioning Translational Medicine, Xuanwu Hospital, Capital Medical University, Beijing, China

## Abstract

**Methods:**

This was a retrospective analysis in a general hospital emergency department in Beijing, China. 212 adult AIS patients treated with thrombolysis who failed to use EMSs were included. In addition to DNT, door-to-vein open time (DVT), door-to-blood sample deliver time (DBT), and 7-day NIHSS scores were evaluated.

**Results:**

137 (64.6%) patients were in the triage nurse-activated group and 75 (35.4%) patients were in the doctor-activated group. The DNT of the triage nurse-activated group was significantly reduced compared with the doctor-activated group (28 (26, 32.5) min vs. 30 (28, 40) min, *p*=0.001). DNT less than 45 min was seen in 95.6% of patients in the triage nurse-activated group and 84% of patients in the doctor-activated group (*p*=0.011, OR 3.972, 95% CI 1.375–11.477). In addition, DVT (7 (4, 10) min vs. 8 (5, 12) min, *P*=0.025) and DBT (15 (13, 21) min vs. 19 (15, 26) min, *p*=0.001) of the triage nurse-activated group were also shorter than those of the doctor-activated group (*p* < 0.05). The 7-day NIHSS scores were not statistically different between the two groups.

**Conclusions:**

Triage nurse-activated urgent emergency evaluation could reduce the door-to-needle time, which provides a feasible opportunity to optimize the emergency department service for AIS patients who failed to use emergency medical services.

## 1. Introduction

Ischemic stroke is one of the leading causes of mortality and disability in China [1, 2]. Intravenous thrombolysis has become a crucial treatment for acute ischemic stroke during the past two decades [3–7]. Data show that earlier reperfusion therapy performance leads to more salvaged brain tissue [8–10]. 1.9 million neurons are lost every minute after an ischemic stroke, which demonstrated that even a small reduction in treatment time may have great benefit to patients' prognosis [11]. Door-to-needle time (DNT) is defined as the time interval from hospital arrival to the onset of the pharmacological (tissue plasminogen activator) infusion, which has been strongly associated with a lower risk of hemorrhagic transformation, mortality, and better functional outcomes at 3 months [12, 13]. A recent study also found an association between shorter DNT and long-term lower all-cause mortality and readmission at one year [14]. Thus, it is critical to explore approaches to reduce DNT to ensure patients receive reperfusion therapy as rapidly as possible.

Currently, several approaches have been reported to reduce DNT [15]. The use of emergency medical services (EMSs) system was independently associated with earlier emergency department (ED) arrival, quicker ED evaluation, and more rapid treatment, which also shortens the DNT [16]. However, only about 59% of all stroke patients acquire EMSs [17]. As per protocol, suspected stroke patients arriving via EMSs would be preliminarily assessed by the in-clinic ED neurologist immediately after hospital arrival. The emergency evaluation was initiated by the multicomponent hospital stroke team if patients met eligibility. Nevertheless, patients who were presented directly to the ED without EMSs would have a waiting period between the triage and preliminary assessment performed by neurologists in the clinic. As a result of the waiting period, postponed initiation of the emergency evaluation performed by the hospital stroke team could contribute to a delay in reperfusion treatment, especially for patients with mild symptoms.

Since triage is the first step for patients who arrive at the ED without EMSs, there is an opportunity for professionally trained triage nurses to directly assess patients and activate the stroke team, theoretically reducing the time until neurologist evaluation in the ED clinic. This study aimed to determine whether triage nurse-activated emergency evaluation would reduce the DNT.

## 2. Materials and Methods

### 2.1. Study Design and Setting

This was an observational retrospective cross-sectional study and was carried out in the emergency department (ED) of Xuanwu Hospital in Beijing from January 2019 to December 2019. This hospital has set a stroke center at the ED to provide emergency evaluation for suspected stroke patients and stroke units to provide comprehensive management for patients with a final diagnosis of stroke. The emergency evaluation was carried out by the hospital stroke team which mainly composed of neurologists and neurosurgeons and depended on multidisciplinary cooperation among the emergency department, intervention center, radiology department, laboratory department, and vascular ultrasound department. Suspected stroke patients were accompanied by the stroke team throughout assessment, examination, and treatment.

### 2.2. Participants

Acute ischemic stroke (AIS) patients diagnosed by computed tomography (CT) or magnetic resonance imaging (MRI) who received emergency evaluation services at ED were screened in this study. Eligible patients were aged ≥18 years and accepted intravenous thrombolysis with informed consent. The exclusion criteria are as follows: (1) patients transported by EMSs; (2) patients with laboratory and/or imaging examinations at other hospitals; and (3) patients with incomplete clinical data. A total of 212 AIS patients were finally included in this study and divided into two groups according to the type of personnel who initiated the urgent emergency evaluation service. 137 patients received the urgent emergency evaluation, activated by triage nurses, and 75 patients were activated by doctors (Figure 1).

### 2.3. Procedure

Procedure of the doctor-activated group: in the doctor-activated group, nurses triaged suspected stroke patients to a higher visit grade and priority if they presented within 4.5 hours of symptom onset or at a time when patients were known to be well by themselves. Doctors in the Neurology Clinic of the emergency department then performed a preliminary examination and assessment and activated the hospital stroke team if patients met eligible criteria. In the meantime, the disease severity of suspected stroke patients would be evaluated by the stroke team as ED nurses insert an indwelling catheter to collect and send blood samples for examination. Subsequently, the radiology department would be contacted to perform a head CT scan for definitive diagnosis. Under the cooperation of the stroke team and emergency department personnel, intravenous thrombolysis therapy was performed in the emergency room for patients who met the indications of intravenous thrombolysis and completed informed consent.

Procedure of the triage nurse-activated group: 6 nurses cooperated with the study and were designated as triage nurses. The criteria for triage nurses were as follows: (1) emergency specialist nurses with more than 5-year work experience; (2) nurses with a bachelor's degree or above; (3) nurses with 3 months of clinical practice in cerebrovascular units; and (4) nurses who were trained in the process of stroke rescue, with solid theoretical knowledge and practical skills in stroke care. They were also trained to master the fast diagnosis of AIS to acquire certification. The 6 triage nurses would directly participate in the evaluation, treatment, and transport of the suspected AIS patients. Triage nurses would first measure vital signs and evaluate suspected stroke patients using the Face-Arm-Speech-Time (FAST) scale, which includes sudden face numbness or weakness, arm(s) numbness or weakness, and slurred or hard-to-understand speech. Triage nurses would then directly initiate the emergency evaluation implemented by the hospital stroke team if the patient suffered any of the above symptoms and the time from symptom onset was within 4.5 hours [18]. The subsequent procedure of treatment was the same as the doctor-activated group (Figure 2).

### 2.4. Data Collection

Patients' general demographic information, route of transportation to the ED (visit on their own or transfer by ambulance), prehospital call (yes or no), and time of visit were collected by exporting from the triage system. The time metrics were recorded by filling in the self-made “Emergency Evaluation Form for Stroke Patients,” including the patient's arrival, venipuncture, blood sample delivery, and the onset of the pharmacological infusion. Disease condition and prognosis information including scores of the 7-day National Institute of Health Stroke Scale (NIHSS) was also evaluated by physicians of the hospital stroke team.

The accuracy rate of triaging-possible AIS patients is referred to as the proportion of patients with definitive AIS among all patients who received emergency evaluation services from the hospital stroke team.

In addition, DNT is defined as the time interval between when the patient enters the ED and the onset of pharmacological (tissue plasminogen activator) infusion; door-to-vein open time (DVT) is defined as the time interval from patients entering the ED to indwelling needle puncture completion; and door-to-blood sample delivery time (DBT) is defined as the time interval from patients entering the ED to the reception of the blood sample in the clinical lab.

### 2.5. Statistical Analysis

The constituent ratios of variables such as sex, the route of transportation to the ED, prehospital call, and visit time were compared using Chi-squared tests. Variables with normal distributions were presented as mean ± SD and were tested for significance using an independent *t*-test. Variables with skewed distributions such as time metrics, scores of NIHSS, and 7-day NIHSS were presented as medians (*P*_25_ and *P*_75_) and compared using the Mann–Whitney *U* test. The accuracy rate of triaging-possible AIS patients among two groups was compared using Chi-squared tests. We considered *P* values less than 0.05 as statistically significant. Multiple analysis was performed using logistic analysis. All statistical analyses were conducted using Software Statistical Product and Service Solutions (SPSS) Version 23.0.

## 3. Results

A total of 840 suspected stroke patients without EMSs were screened, with 554 and 286 patients activated by triage nurses and doctors, respectively. There were no significant differences between the two groups with the accuracy of finally diagnosing stroke patients (triage nurse-activated group: 83.9% vs. doctor-activated group: 85.7%, *P*=0.291).

### 3.1. Baseline Characteristics of Patients

A total of 212 AIS patients accepted intravenous thrombolysis and were included in this study, of whom 137 (64.6%) received triage nurse-activated emergency evaluation. The age of all participants ranged from 20 to 97 years. The mean age of the triage nurse-activated group was 61.20 ± 11.75 years, and 73.0% of participants were male. There was a median NIHSS score of 5.

There was no significant difference between the two groups with regard to the distribution of sex, visit time (*P* > 0.05), average age (*P* > 0.05), and median score of NIHSS (*P*=0.094), and detailed data are listed in Table 1.

### 3.2. Door-to-Needle Time in Two Groups

DNT of the triage nurse-activated group was significantly reduced compared with the doctor-activated group (28 (26, 32.5) min vs. 30 (28, 40) min, *P*=0.001). In addition, DVT (7 (4, 10) min vs. 8 (5, 12) min, *P*=0.025) and DBT (15 (13, 21) min vs. 19 (15, 26) min, *P*=0.001) in the triage nurse-activated group were also shorter than those in the doctor-activated group (Table 2).

After adjustment for age, sex, and the severity of stroke, DNT less than 45 min was seen in 95.6% of patients in the triage nurse-activated group and 84% of the other group (*P*=0.011, OR 3.972, 95% CI 1.375–11.477), which indicated that triage nurse-activated emergency evaluation was strongly associated with DNT less than 45 min (Table 3).

### 3.3. 7-Day NIHSS Score

There was no significant difference in median 7-day NIHSS scores between the two groups (case group: 2 vs. control group: 1, *P*=0.893).

## 4. Discussion

This retrospective study revealed that triage nurse-activated urgent emergency evaluation could significantly reduce DNT as well as DVT and DBT with comparable accuracy of final diagnosis among stroke patients with doctor-activated emergency evaluation. In addition, nurse-activated emergency evaluation of the hospital stroke team was strongly associated with DNT less than 45 minutes.

Since intravenous thrombolysis has proven effective for acute ischemic stroke (AIS) patients [19, 20], the association between shorter DNT and a better functional outcome has been widely explored [3, 4]. In addition to better short-term functional outcomes, a recent study published in JAMA revealed that shorter DNT was also correlated with better long-term outcomes and each 15-minute increase in DNT was distinctively associated with higher all-cause mortality within 90 minutes after ED arrival [14]. Thus, it is pivotal to reduce DNT for better functional outcomes. EMSs have been reported to be an effective prehospital strategy to reduce the time metrics of stroke treatment. However, many patients still failed to use EMSs. Other promising in-hospital opportunities to reduce DNT still need to be explored for patients who do not use EMSs.

As the first contact medical personnel and the whole-process manager of stroke patients, nurses perform a vital role in evaluation, diagnosis, and treatment [21, 22]. Recent studies have demonstrated the effectiveness of nurses in the treatment of stroke patients [22]. A nurse-led stroke team implementation may be an effective method for improving time-sensitive metrics of stroke care and increasing institutional compliance with recommended national guidelines [23]. Furthermore, improving the ability to recognize and care for stroke patients by more specific training in stroke nurses is an important factor, which can reduce the delay of intravenous thrombolysis in the hospital and help expedite AIS-presenting patients' arrival to the hospital after stroke [24]. In our study, nurse-activated emergency evaluation decreased  DNT  as well as other time metrics of treatment for AIS patients.

The benchmark of DNT was set at 60 minutes by some guidelines [25, 26], yet Man et al. indicated that patients that accepted IVT whose DNT was less than 45 minutes had the lowest mortality and readmission rates [14]. Therefore, in our study, we also revealed a significant association between nurse-activated emergency evaluation and the DNT within 45 minutes, which further clarified the efficacy of nurse-activated emergency evaluation. Recently, hospitals have set a DNT goal within 60 minutes for at least 75% of patients and a DNT within 45 minutes for at least 50% of patients [27, 28]. In our study, the proportion of patients with DNT less than 45 minutes had reached 95.6% in the triage nurse-activated group.

Hence, implementation of triage nurse-activated emergency evaluation achieved elimination of the waiting period between triage and clinical reception with advancement of the evaluation and diagnosis of stroke patients in the meantime. The score of 7-day NIHSS had no significant difference between the two groups in our study, which may be due to the small sample size and short-term follow-up. And, our results showed male gender was negatively associated with DNT less than 45 min, which may also be due to the selection bias brought by the small sample size.

The successful implementation of nurse-activated emergency evaluation depends on experienced triage nurses and suitable tools in stroke recognition. The lack of knowledge and ability of triage nurses were one of the critical factors for the delay in the treatment of stroke patients [29]. It is crucial for a qualified triage nurse to have the clinical acumen and recognition of complicated conditions, strong organization skills, and proficient management and coordination abilities. Strict admittance requirements and standardized training are effective measures to guarantee the ability of triage nurses. In our study, the triage nurses were well-trained for stroke recognition, assessment, and treatment. The recognition of stroke was the first and most pivotal step for suspected AIS patients [30]. Numerous stroke recognition instruments have been developed for EMS and ED personnel to improve the sensitivity and specificity of identification [31]. The FAST scale has been reported as one of the triage protocols in reducing door-to-CT time and DNT in patients who presented directly to the ED, which has an extremely high sensitivity for stroke recognition when used by paramedics [32, 33]. Besides, the FAST scale is easy to use and boasts a 76.9% sensitivity and a 69.4% specificity of identification for community-dwelling mild stroke patients [34]. In our study, the accuracy of diagnosing stroke patients in the triage nurse-activated group was comparable to that of the doctor-triage group.

We made great efforts focused on the elimination of the delay between triage and neurologist-performed preliminary assessment for suspected stroke patients. Our study also indicated that stroke nurses have an indispensable effect on the ED management of stroke patients. An increasing number of countries and regions have implemented stroke nurses in the ED to provide patients with whole visit services [22, 35]. Stroke nurses are not only practitioners of medical advice but also serve as managers, coordinators, and leaders of thrombolytic procedures. Stroke nurses participating in the treatment of stroke patients in the ED would increase the rescue efficiency and improve the prognosis of patients [36]. Finally, our study also provides a reference for the establishment of nurse-led stroke teams in China.

## 5. Limitations and Future Directions

The single source, limited size of the sample, and short period of data collection limit the statistical power of this study and the generalizability of the study results. The outcomes of AIS patients were limited by 7-day NIHSS scores without observing the outcomes of 90 days or longer. The results of our study should be tested in a multicenter study with a larger sample size in the future. Future studies may also focus on extending the study period and increasing the evaluation indexes.

The remaining opportunity for improving stroke management involves advancing triage to prehospital treatment by establishing a mobile stroke unit focused on providing whole stroke management, including prehospital, in-hospital, and posthospital treatment. Finally, the integration of screening, treating, and rehabilitation by interdisciplinary care teams is an integral area of study to facilitate quality improvement of ED services.

## 6. Conclusion

The emergency evaluation services activated by triage nurses would shorten the time of treatment for AIS patients based on comparable accuracy of recognition with neurologists in the ED clinic in this study, which provides a feasible opportunity to optimize the emergency department service for AIS patients who failed to use emergency medical services.

## Figures and Tables

**Figure 1:** Screening flowchart of participants.

**Figure 2:** Procedure of the doctor-activated or nurse-activated group.

**Table 1:** Baseline patient characteristics.

	Triage nurse-activated, *n* = 137	Doctor-activated, *n* = 75	*P* value
Male (%)	73.0	72.0	0.873
Age (yr)	61.20 ± 11.75	63.99 ± 11.40	0.094
Visit time			
2am to 8am	15	6	0.591
8am to 5pm	62	39	
5pm to 2am	60	30	
NIHSS			
Median (*P*_25_, *P*_75_)	5 (4, 7)	4 (3, 7)	0.094

**Table 2:** Outcome indicators in two groups.

Outcome indicators	Triage nurse-activated, *n* = 137	Doctor-activated, *n* = 75	*P* value
DNT	28 (26, 32.5)	30 (28, 40)	0.001
DVT	7 (4, 10)	8 (5, 12)	0.025
DBT	15 (13, 21)	19 (15, 26)	0.001
7-day NIHSS	2 (0, 4)	1 (0, 5)	0.893
Patients with DNT less than 45 min	131	63	0.004

**Table 3:** The association between nurse-activated emergency evaluation and DNT less than 45 min.

	Adjusted OR	95% CI	*P*
Nurse-activated emergency evaluation	3.972	1.375–11.477	0.011
Age	0.971	0.925–1.018	0.225
Male	0.268	0.096–0.752	0.012
NHISS	0.993	0.901–1.094	0.887

## Data Availability

All supporting data are included within the article.
